# Factors predicting surgical site infection after posterior lumbar surgery: A multicenter retrospective study

This article has been retracted.

**DOI:** 10.1097/MD.0000000000006042

**Published:** 2017-02-03

**Authors:** Tao Wang, Hui Wang, Da-Long Yang, Li-Qiang Jiang, Li-Jun Zhang, Wen-Yuan Ding

**Affiliations:** a Department of Spinal Surgery, The Third Hospital of Hebei Medical University, Shijiazhuang; b Department of Orthopaedics, HanDan Central Hospital, HanDan; c Department of Orthopaedics, The First Hospital of Shijiazhuang, Shijiazhuang, China.

**Keywords:** factors, posterior lumbar surgery, surgical site infection

## Abstract

This is a retrospective study.

The purpose of this study is to explore incidence and risk factors for surgical site infection (SSI) after posterior lumbar surgery.

SSI is a common complication after posterior lumbar surgery, bringing mental and physical pain and prolonging hospital stay. However, predisposing factors, as reported less, remain controversial.

Patients who underwent posterior lumbar surgery at 3 centers between 2006 and 2016 were included. The possible factors include 3 aspects: demographic variables-age, sex, body mass index (BMI), waist-to-hip radio (WHR), hypertension, diabetes, heart disease, smoking, drinking, steroidal injection, surgical time between June and September, preoperative shower; blood test variables-white blood cell (WBC), neutrophil, red blood cell (RBC), hemoglobin (Hb), total protein (TP), albumin, albumin/globulin (A/G), C-reactive protein (CRP), procalcitonin (PCT), erythrocyte sedimentation rate (ESR) and surgical related variables-operation time, blood loss, operative level, instrumentation, incision length. Factors related with SSI were also performed by multivariate analysis.

The prevalence of SSI was 3.00% (267 cases of 8879) had a postoperative wound infection. There were significant difference in WHR (0.92 vs 0.83), WBC (4.31 vs 6.69), TP (58.7 vs 65.2), albumin (36.9 vs 43.2), CRP (2.01 vs 0.57), PCT (0.097 vs 0.067), operation time (217.9 vs 195.7), blood loss (997.1 vs 915.3) and operative level (3.05 vs 2.45) and incision length (24.1 vs 20.0) between SSI group and non-SSI group. >60 years old, female, BMI <18.5 and >30.0, diabetes, male smoking, preoperative steroidal injection, surgical time between June and September, no preoperative shower, instrumentation surgery were risk factors for SSI after posterior lumbar surgery.

Many factors, >60 years old, female, BMI, WHR, diabetes, male smoking, preoperative steroidal injection, surgical time between June and September, preoperative shower, WBC, TP, albumin, CRP, PCT, operation time, blood loss and operative level, instrumentation surgery and incision length, could predict SSI after posterior lumbar surgery. Measure should be taken before surgery to lower incidence of SSI after surgery.

## 1 Introduction

Surgical site infections (SSI), serious complication after posterior lumbar surgery, are a hospital-acquired infection of the skin, soft tissue, or bone, which may cause severe morbidity with poor quality of life and even risk for life. Mentioned above would lead to unfavorable surgical outcomes, extend length of hospital stays, and increase costs.^[1–5]^ Some studies reported that incidence for SSI after spinal surgery was between 0.7% and 12% depending on the operative type and the studied population.^[6–10]^

Bryan^[11]^ studied on SSI and held that female patients, inpatient status, insulin-dependent diabetes, using preoperative steroid more than 10 days, hematocrit < 35, BMI >30, wound class, ASA class and operative duration were risk factors for SSI. Nevertheless Klemencsics^[12]^ considered older age, higher BMI, diabetes, ischemic heart disease, arrhythmia, chronic liver disease, and autoimmune disease as the risk factors for SSI. The factors increased incidence of SSI remains controversial.

The purpose of our study is to assess prevalence and explore risk factors of SSI by *t* test and multivariate analysis.

## 2 Materials and methods

### 2.1 Ethics statement

This is approved by Ethics Committee of Third Hospital of HeBei Medicle University, the First Hospital of Shijiazhuang and HanDan Central Hospital.

### 2.2 Patients

Two hundred sixty-seven patients with infection and 8612 patients without infection after posterior lumbar were included in our study from the Third Hospital of HeBei Medicle University (140 patients with SSI of total 4655 patients, 3.0%), the First Hospital of Shijiazhuang (58 patients with SSI of total 1964 patients, 2.9%), and HanDan Central Hospital (69 patients with SSI of 2260 total patients, 3.1%). from January 2006 to November 2016. The inclusion criteria: ≥20 years old; suffer from lumbar disc herniation, stenosis, or inflammation; patients who underwent posterior lumbar surgery. The exclusion criteria were as follows: have history of any spinal surgery before this surgery; have spinal deformities (including scoliosis, sacralization, or lumbarization); have spinal trauma or tumors; arthropathy in the lower limbs.

### 2.3 Variables

We analyzed possible factors including 3 aspects: demographic variables-age, sex, BMI, WHR, hypertension, diabetes, heart disease, smoking, drinking, steroidal injection, surgical time between June and Sep, preoperative shower; blood test variables-WBC, neutrophil, RBC, Hb, TP, albumin, A/G, CRP, PCT, ESR and surgical related variables-operation time, blood loss, operative level, instrumentation, incision length.

The methods were carried out in accordance with the approved guidelines. Two authors identified and collected all the data of patients according to inclusion criteria and exclusion criteria. In addition, 2 authors were responsible for data analyses. All measurement data are presented as the mean ± SD (standard deviation) when data satisfied criteria for normality with *P* > 0.05. Measurement data like age, BMI, WHR, WBC, neutrophil, RBC, Hb, TP, albumin, A/G, CRP, PCT, ESR, operation time, blood loss, operative level, incision length satisfied criteria for normality and homogeneity of variance, statistical analysis between groups was performed using independent samples *t* test. And count data, like sex (male/female), hypertension, diabetes, heart disease, smoking, drinking, steroidal injection, surgical time between June and September, preoperative shower, instrumentation, *χ*^2^ test were used for data analysis. The Kolmogorov–Smirnoff test was used to verify the normal data distribution. Statistical significance levels were considered to be *P *< 0.05. All statistical analyses were carried out using SPSS, version 21.0 (SPSS Inc, Chicago, IL).

## 3 Results

As for demographic variables, age (66.1 ± 8.6) and WHR (0.92 ± 0.83) for SSI group were significantly larger than these for non-SSI group (57.7 ± 12.1, 0.83 ± 0.75, respectively), as shown in Table 1. Additionally, we found in Table 1 that female patients, male patients with smoking, patients with diabetes, preoperative steroidal injection, surgery between June and September, and without preoperative shower were more likely to suffer from infection after posterior lumbar surgery.

**Table 1:** Variables between 2 groups.

Table 1 shows that no significant difference in neutrophil, RBC, Hb, A/G, ESR between 2 groups were noticed. WBC (4.31 ± 0.54), TP (58.7 ± 4.4), and albumin (36.9 ± 3.2) for SSI group were significantly smaller than these for non-SSI group (6.69 ± 1.15, 65.2 ± 3.5, 43.2 ± 3.5, respectively), however, CRP (2.01 ± 0.69) and PCT (0.097 ± 0.038) for SSI group were significantly larger than these for non-SSI group (0.57 ± 0.32, 0.067 ± 0.030, respectively).

In Table 1, operation time (217.9 ± 20.6), blood loss (997.1 ± 114.5), operative level (3.05 ± 1.26), and incision length (24.1 ± 1.8) for SSI group were significantly larger than these for non-SSI group (195.7 ± 18.8, 915.3 ± 60.6, 2.45 ± 0.95, 20.0 ± 1.8, respectively). We found that patients with instrumentation were more likely to suffer from infection.

Moreover, we performed multivariate analysis, indicating that female patients, patients who >60 years old, BMI <18.5 and >30.0, larger WHR, diabetes, smoking male, preoperative steroidal injection, surgical time between June and September, no preoperative shower, relatively low WBC, TP and albumin, relatively high CRP and PCT, more operation time, blood loss and operative level, instrumentation and larger incision length were easier to have infection after posterior lumbar surgery (Tables 1 and 2).

**Table 2:** Factors by multivariate analysis between 2 groups.

## 4 Discussion

The prevalence of SSI is one of the most common complications after spinal surgery, was 4.3% in 1532 patients as reported by Lee.^[10]^ SSI have a serious influence on patients’ life quality when these occur. Cost of treatment, increased hospital stay, and increase of the need for rehospitalization are huge burden for families and even for society. The previous study^[12]^ reported that $1.6 billion was used for treatment of SSI annually. The aim of our study is to explore the incidence and risk factors for SSI after posterior lumbar surgery. Risk factors for SSI were reported in the previous study: obesity (BMI), longer operation time, diabetes mellitus, smoking, history of previous SSI, and type of surgical procedure.^[4]^ Our large, multicenter study showed that incidence of SSI after posterior lumbar surgery was 3% (267 of 8879). And the incidence for male patients, female patients, and patients with diabetes, male smoking, preoperative steroidal injection, surgical time between June and September and without preoperative shower were 1.1%, 4.7%, 5%, 1.7%, 34%, 4.8%, 0.6% respectively. Female patients, patients >60 years old, BMI <18.5 and >30.0, patients with larger WHR, diabetes, smoking male, preoperative steroidal injection, surgical between June and September, without preoperative shower, patients who have relatively low WBC, TP and albumin, relatively high CRP and PCT, more operation time, blood loss and operative level, instrumentation surgery and larger incision length as our results indicated were risk factors for SSI after posterior lumbar surgery.

In our study, female patients, patients who >60 years old, BMI <18.5 and >30.0, patients with larger WHR, diabetes, smoking male, preoperative steroidal injection, surgical time between June and September, without preoperative shower were significant risk factors for SSI after posterior lumbar surgery. Results revealed that older age was a factor markedly affecting SSI and multivariate analysis further identified that patients >60 years old was a real factor for SSI. Relatively poor health status and immune system should be the reasons. Diabetes was not a significant risk factor as reported in few studies.^[13,14]^ We regarded it as an important risk factor for SSI, which was the same with most studies.^[6,9–11]^ Decreased local tissue perfusion is caused by diabetic microangiopathy, which could cause impaired granulocyte function due to the impaired platelet-derived growth factor function. Though BMI in 2 groups were similar by *t*-test analysis, multivariate analysis showed that both BMI <18.5 and >30 were risk factors for SSI. The former literature^[15]^ only considered BMI >30 as a risk factor. BMI <18.5 indicated that patients have a relatively poor nutritional status. We also found significantly larger WHR in SSI group, implying abdominal obesity in SSI group. Interestingly, patients operated between June and September and without shower within 3 days before operation were easier to suffer from SSI. The average air temperature between June and September in Shijiazhuang and HanDan districts was more than 30°C, in which it was beneficial to bacterial reproduction.

Improving Hb to >11 g/L and TP > 60 g/L could lower incidence of SSI.^[13]^ But in our study, level of Hb had no remarkable relation to SSI, but relatively low WBC, TP, and albumin were closely related to SSI after surgery. It was well known that WBCs as defence soldiers protect our body from virus or bacteria. Even though the level of WBC is within normal limitation in the SSI group, but the relatively low level implied relatively poor immune ability when virus or bacteria invade the body. In the same way, relatively low TP and albumin indicated patients in relatively poor nutritional status, which had poorer ability to prevent our body from virus or bacteria than those in good nutritional status. CRP and PCT are commonly used detection index of inflammation, we just checked preoperative CRP and PCT and found that CRP and PCT in SSI group were markedly higher than these in non-SSI group. The reason remains unclear.

We also compared surgical-related variables between SSI and non-SSI groups. Our results showed that operation time was 217.9 minutes in SSI group, which is markedly larger than that in non-SSI group (195.7 minutes). Operation time was regarded as a biggest risk factor for SSI previously.^[16]^ We considered the surgical levels as a biggest risk factor for SSI after surgery. More surgical levels increase the risk of SSI implying that surgery needed more operation time, more blood loss, more blood transfusion, and larger incision length. Surgery with instrumentation increased incidence of SSI after posterior lumbar surgery, compared with surgery without. Surgery with instrumentation indicated that we need longer surgical procedures and more operation time, which may lead to increased duration of tissue traction, higher risk of ischemic necrosis, and wound contamination. Measures, washing with >2000 mL of normal saline for operation field, irrigation of the wound, and loosening of wound tension for reducing risk of SSI related to surgical variables should be taken.^[16,17]^

The present study has several limitations. First, it was a retrospective study, we need to conduct a prospective study to further explore the risk factors for SSI after posterior lumbar surgery; second, some factors could not be observed due to retrospective study, for example, whether improving TP and albumin to normal level before surgery could reduce risk of SSI or not; relation between subcutaneous fat thickness and SSI; operating room is closed or not during surgery; how many doctors in operative room, and so on; third, data on microbiology was not analyzed due to lack of related data or incomplete data.

However, even though it has these limitations, large-scale and multicenter study is valuable for surgeons to notice some variables leading to SSI before surgery.

In conclusion, our multicenter study found that multipaths and diverse factors could cause SSI and female patients who >60 years old, BMI <18.5 and >30.0, patients with larger WHR, diabetes, smoking male, preoperative steroidal injection, surgical time between June and September, relatively low WBC, TP and albumin, relatively high CRP and PCT, more operation time, blood loss and operative level, without preoperative shower, instrumentation surgery and larger incision length could significantly increase risk of SSI. Preoperative counseling and intervention, along with targeted treatment strategies for a specific set of risk factors, may decrease the rate of SSI. A prospective study is needed to assess factors for SSI after posterior lumbar surgery.
